The article "Hybrid Composite Laminates Reinforced with Kevlar/Carbon/Glass Woven Fabrics for Ballistic Impact Testing" was published in 2014. Journal: ScientificWorldJournal.

# Hybrid Composite Laminates Reinforced with Kevlar/Carbon/Glass Woven Fabrics for Ballistic Impact Testing

**DOI:** 10.1155/2014/413753

**Published:** 2014-05-12

**Authors:** Elias Randjbaran, Rizal Zahari, Nawal Aswan Abdul Jalil, Dayang Laila Abang Abdul Majid

**Affiliations:** Department of Aerospace Engineering, Faculty of Engineering, Universiti Putra Malaysia, 43400 Serdang, Selangor Darul Ehsan, Malaysia

## Abstract

Current study reported a facile method to investigate the effects of stacking sequence layers of hybrid composite materials on ballistic energy absorption by running the ballistic test at the high velocity ballistic impact conditions. The velocity and absorbed energy were accordingly calculated as well. The specimens were fabricated from Kevlar, carbon, and glass woven fabrics and resin and were experimentally investigated under impact conditions. All the specimens possessed equal mass, shape, and density; nevertheless, the layers were ordered in different stacking sequence. After running the ballistic test at the same conditions, the final velocities of the cylindrical AISI 4340 Steel pellet showed how much energy was absorbed by the samples. The energy absorption of each sample through the ballistic impact was calculated; accordingly, the proper ballistic impact resistance materials could be found by conducting the test. This paper can be further studied in order to characterise the material properties for the different layers.

## 1. Introduction

During the life of a structure, impacts by foreign objects could be expected to occur during manufacturing, service, and maintenance operations. An example of in-service impact occurs during aircraft takeoffs and landings when stones and other small debris from the runway were propelled at high velocities by the tires. During the manufacturing process or during maintenance, tools could be dropped on the structure. In this case, impact velocities are small but the mass of the projectile is larger. Laminated composite structures are more susceptible to impact damage than a similar metallic structure. In composite structures, impacts create internal damage that often cannot be detected by visual inspection. This internal damage can cause severe reductions in strength and can grow under load. Therefore, the effects of foreign object impacts on composite structures must be understood, and proper measures should be taken in the design process to account for these expected events. Concerns about the effect of impacts on the performance of composite structures have been a factor in limiting the use of composite materials. For these reasons, the problem of impact has received considerable attention in developing not only technical know-how but also a practical and analytical approach to problem solving that can allow addressing a range of aerospace engineering challenges. This was particularly true under high velocity ballistic impact scenarios [1].

The body of aircrafts is susceptible to accidental damages from low- to high-energy impacts of such hazards as dropped tools during maintenance, runway debris, hailstones, and sandstorm. These impacts could bring about considerable strength reduction, and the localized damage was potentially a source of mechanical weakness, particularly under the mechanical applications [2–4].

Furthermore, the damage consequent upon a minor impact can grow to large size under the mechanical applications. The nature of the impact damage in hybrid composite laminates ranges from surface damage and subsurface damage to complete penetration, depending upon the impact loading conditions. Generally, under the ballistic impact, impact loading on composite laminates can cause surface or internal damage in the form, including fibre breakage, delamination, and matrix cracking. Such damages can reduce laminate tensile strength, resulting in so-called part through the thickness damage. This sort of damage is of a complicated form, consisting of fluctuating amounts of matrix cracks, fibre cracks, and delamination. The complexity of the damage makes it difficult to assess the precise mechanisms controlling strength reduction. Among these modes of impact damage, delamination has the most detrimental effects on laminate stiffness and strength and has received a considerable amount of attention [5–9]. High velocity impact involves projectiles moving at higher velocities such that the local target materials behave like fluids, and the stress induced by the impact is many times the material strength. The goal for this classification is the energy transfer in the middle projectile and target; energy waste and damage propagation mechanisms withstand extreme transfiguration as the velocity of the projectile changes. One of the possible ways of magnifying the ballistic limit is to employ textile composites. The kinetic energy of the projectile once impacted into the target is scattered and absorbed in various lanes by the target. The main energy-absorbing mechanisms throughout the ballistic impact include kinetic energy absorbed by the moving pellet on the back face of the target, energy absorbed due to tensile failure of the primary fibers' layer, energy absorbed due to the elastic deformation of the secondary fibers' layer, energy absorbed due to matrix cracking and delamination, and frictional energy absorbed in the course of penetration. At high velocity or ballistic impact, the response of the structural element is governed by the local behaviour of the material in the region of the impacted zone; the impact response of the element is generally independent of its assist conditions. The contact cycle of the impact is smaller than the time cycle of the lowest vibration mode of the structure. Hyperimpact involves projectiles moving at extremely high velocities such as the local target materials behaving like fluids, and the stress induced by the impact is many times the material strength [10].

Sultan et al. [9] mentioned that, as the plate specimen thickness continued to increase, the damage on the lower skin slightly decreased, which could not be seen. In addition, as the plate thickness increased, the maximum impact load and impact energy increased relatively. Impact damage was in the form of perforation, fibre breakage, and matrix cracking. In the current study, the effects of stacking sequence layers of hybrid composite materials in energy absorption under the high velocity ballistic have been investigated. Impact specimens in terms of composite structures consisting of Kevlar, glass, and carbon fabrics and epoxy layers with different sequences were fabricated via hand lay-up method.

## 2. Manufacturing Procedure

### 2.1. Materials

Three types of fibres, including glass, carbon, and Kevlar, were used in fabricating the specimens. The Kevlar fabric used in all composite target constructions was plain-woven Hexcel Aramid (polyparaphenylene terephthalamide), high-performance fabric Style 706 (Kevlar KM-2, 600 denier) with a real density of 180 g/m^2^. Room temperature curing and the ratios of 50 parts epoxy resin (EPOKUKDO YD-128) to 50 hardeners (Polyamide-Domide (A.V: 350)) by weight were comprehensively cured after seven days at 20°C [11, 12].

Table 1 illustrates the ordering and sequence of fibres plies in each hybrid composite materials. As mentioned in the literature review, when loads are parallel to the fibres (0°), the ply is much stronger and stiffer than whereas loads are transverse (90°) to the fibre direction. Therefore, the ply orientation is (0°), the thickness of all is 1.78 mm, and the density of all the hybrids is about 1.7 g/cm^3^.

### 2.2. Experimental Testing Procedure

The specimens were produced by hand lay-up method. The experimental setup was according to guidelines given in the NIJ Standard 0108.01 [10], shown in Figure 1. Compressed Helium gas was used as the working fluid. The air pressure from the compressor was kept constant at 0.6 × 10^3^ kPa while Helium pressure was increased from 1.4 × 10^3^ kPa to 4.1 × 10^3^ kPa. However, the gun tunnel can be operated at maximum of 21 × 10^3^ kPa. The air pressure was used to open the Helium gas valve at the gun tunnel barrel after its trigger was pushed. The gun tunnel barrel length is about four meters measured from the pellet reload section and a test section chamber was placed at the end of the gun tunnel barrel. Test section is made of high strength steel that give out most protection during the experiment. The test section chamber is 600 × 450 × 450 mm^3^ in length, height, and width, respectively, as shown in Figures 2 and 3 [13–15]. It gives enough space for the pellet to be calibrated and stopped. The trigger for the gun tunnel is the places near the pellet reload section where it is far away from the test section chamber making much safety in working area and also Figures 2 and 3 display the actual gun tunnel used for the experiment.

Figure 4 shows the schematic of the mild steel pellet being used in the experiment. Cylindrical pellets were used in the experiment to calibrate the pellet speed by varying Helium gas pressure. Pellet used in the experiment was made of mild steel with 6.75 g of weight. The length is 13.07 mm by 8.48 mm in diameter. It has a smooth cylindrical surface to possess the minimum friction and drag during its light. Together with that, oil is also being used as a tube to the pellet, which helps to reduce surface friction contact.

### 2.3. Calculation of Velocity

This invention relates to high-speed cameras and in particular to high-speed cameras having resolution times of less than one-tenth microsecond. High frame rates required a sensor with good sensitivity, either a very good shuttering system or a very fast strobe light, and also require some means of capturing successive frames, either with a mechanical device or by moving data off electronic sensors very quickly. In such higher frame rates, it is found that a slight difference in debris cloud formation was captured in the interframe of 4 microseconds, which is equivalent to the 250,000 frames per second, and the debris fragment distributions appear to be slightly narrower and thinner at cryogenic temperature.

### 2.4. Calculation of Energy

It is an established fact that absorbed energy by a specimen in ballistic test is means to quantify impact-penetration resistance. Therefore, the absorbed kinetic energy of armor-projectile interaction can be linked by equation for determining kinetic energy.

## 3. Results and Discussion

### 3.1. Ballistic Impact Testing

#### 3.1.1. High-Speed Photography and Calculating the Velocities of the Pellets

After fabricating the required number of specimens, a variety of tests were carried out to investigate the behaviour of the various groups of specimens when they were subjected to impact and then under compression. Moreover, the number of experimental runs is fifty.

Figure 5 shows the process of penetration of pellets into the specimens. In addition, Figure 6 illustrates the amount of ejected materials in all the six different types of specimens, including the five hybrids and the pure carbon fibre that are diverse to each other. The amount of ejected materials is evidence for absorbing energy. The percentage average of weight loss is 9.8%; as a consequence, Hybrid 1 and Hybrid 5 are above the average and the rest of the specimens are below average. If the amount of ejected materials becomes increased, the energy absorption becomes decreased. The amount of ejected materials is a significant evidence for absorbing energy. If the amount of ejected materials increases, the energy absorption will consequently decrease. Therefore, among the hybrid composite materials, the highest amount of ejected materials belongs to Hybrid 1 with 19.84% and the lowest one belongs to Hybrid 2 with 3.54%.

### 3.2. Postimpact Images and Calculating the Perimeter of Impacted Zone

Figure 7 shows all six specimens, including Hybrid 1 to Hybrid 5 and pure carbon fibre, after ballistic impact, that is, postimpact images of damaged specimens' profiles. On the left side, impact-induced damage profile viewed from the front face and, on the right side, impacted damage profile viewed from the back face.  Figure 8 illustrates the approximate values of perimeter of impacted zone in millimeters, which are impacted by the pellets. The close correlation is typically comparative at the level with Hybrid 5 and the difference between them is 0.55 m/s. Additionally, the difference between the maximum and minimum final velocities is 12.51 m/s.

### 3.3. Calculating the Energy Absorption upon the Ballistic Impact

Figure 9 shows the changes in ballistic impact energy absorption of Hybrid 1 to Hybrid 5 and the pure carbon fibre at 182 m/s as an initial velocity. The highest concentration of energy absorption is ranging around 95 joules, from a maximum of 95.17 J to a minimum of 95.01 J, such as Hybrid 2 (95.17 J), Hybrid 4 (95.15 J), Hybrid 5 (95.04 J), and Hybrid 3 (95.01 J). The amounts of energy absorption of Hybrid 2 and Hybrid 4 are close to each other; also the difference between both of them is 0.02 J. One more pair of the Hybrids was approximately at the similar level of ballistic energy absorption. Additionally, there is a strong positive linear relationship between the size of the damage zones and the kinetic energy. If the area is larger, higher amount of ballistic energy will be absorbed. Hybrid 2 has the largest impact-conducted area with 188.5 mm and Hybrid 1 has the smallest with 83.2 mm. The impact-conducted areas of Hybrid 2 and Hybrid 4 are approximately closed together and their difference is 12.1 mm. On the other hand, Hybrid 3 and Hybrid 5, with 2.3 mm difference, nearly are aligned. Regarding the fundamentals of the relationship between the ballistic energy absorption and the impact-conducted areas, Hybrid 2 can absorb the maximum amount of ballistic energy absorption and Hybrid 1 can absorb the minimum. This means that the ratio of the maximum and minimum of the perimeter of the impacted zone, which are impact conducted, is about 44.14%.

Table 2 illustrates a set of experimental data in relation to the sorts of changes, which are the manifestation of the amount of absorbed ballistic energy (in a Joule scale unit) of each of the specimens according to final velocities of each pellet (in meter per second) at 182 m/s as an initial velocity. In general, trends unveiled some variation throughout the figure of the information. Turning to the details, it can be demonstrated that, in Hybrid 2, the minimum final velocity is 4.47 m/s and the maximum final velocity, among the hybrid specimens, is in Hybrid 1 (14.36 m/s). Furthermore, in Hybrid 2 is the maximum energy that could be absorbed (95.17 J), among the hybrid specimens, and the minimum of absorbed energy is in Hybrid 1 (94.36 J).

Figure 10 shows the final velocities of the pellets in six types of specimens, while the initial velocity is 182 m/s. Hybrid 2 demonstrated the reduction of the velocities of the pellets less than the other specimens. Among the hybrid specimens, the final velocities of Hybrid 2, Hybrid 3, Hybrid 4, and Hybrid 5 are close to each other; however, they are not united, and the difference among them is 4.29 m/s. Furthermore, Hybrid 2 and Hybrid 4 are approximately at the level and the difference between them is 0.81 m/s. Likewise, in amount of ballistic energy absorption; there is a negligent difference between Hybrid 3 and 5, which amount is 0.03 J. Hybrid 2 has the maximum ballistic impact energy absorption; in contrast, Hybrid 1 (94.36 J) possesses the minimum ballistic impact energy absorption. Moreover, the disparity between the maximum and minimum ballistic impact energy absorption is 0.81 J.

Figure 10 shows the relationship between that the amounts of ballistic impact energy absorption and the final velocities of the pellets, when the initial velocity of the pellets is 182 meter per second. *X*-axis indicates the final velocity in meter per hour and *Y*-axis indicates the amounts of ballistic impact energy absorption in joules. Six different types of specimens, including Hybrid 1 to Hybrid 5 and the pure carbon fibre, were investigated by conducting the impact test. The most desirable specimen should follow the following characteristics: first, it reduces the final velocities of the pellets to its lowest level; second, it should have absorbed the highest rate of ballistic impact energy. Hybrid 2 and Hybrid 4 demonstrated close behaviour in terms of the final velocity and the energy absorption, whose final velocity difference is 0.81 m/s, and the energy absorption difference is 0.02 J. Besides, Hybrid 3 and Hybrid 5 are showing the same close behaviour, whose velocity difference is 0.55 m/s, and the difference of energy absorption is 0.03 J. It can be concluded that the amounts of ballistic impact energy absorption have increased, whereas the final velocities of the pellets have gone down slightly. Among the hybrids, the strongest one is Hybrid 2 and the weakest one is Hybrid 1. Furthermore, among all of them, the strongest one is Hybrid 2 and the weakest one is the pure carbon fibre.

*The Coefficient of Restitution*. The coefficient of restitution (COR) of striking objects is a fractional value representing the ratio of velocities after and before an impact, taking along the line of the impact. Pairs of objects with COR = 1 collide elastically, while objects with COR < 1 collide elastically. For a COR = 0, the objects effectively “stop” during the striking, not bouncing at all. An object (singular) is often described as having a coefficient of restitution as if it were an intrinsic property without reference to a second object. In this case, the definition is assumed to be with respect to strikes with a perfectly rigid and elastic object [16–18]

(1) $$\begin{array}{c} \text{COR}=\frac{\left(\text{velocity}\;\text{after}\;\text{impact}\right)}{\left(\text{velocity}\;\text{before}\;\text{impact}\right)}. \end{array}$$

Figure 11 demonstrates the COR, shown as a percentage, in the six different types of specimens, including Hybrid 1 to Hybrid 5 and the pure carbon fibre. The *X*-axis indicates the types of the specimens and *Y*-axis indicates the percentage of the COR. Hybrid 2 has a minimum COR and Hybrid 1 (among the hybrids) has a maximum COR. Afterward, the difference between them is 5.43%. An average percentage of the COR is about 4.51%. Hybrid 2, Hybrid 4, and Hybrid 5 are below the average line; consequently, Hybrid 1 and Hybrid 3 are above the average line.

## 4. Conclusions

The results show, first, that Hybrid 2 has the superlative energy absorption of 95.17 J. Second, it can be concluded that stacking the first layer with glass fibre is better than to use the Kevlar fibre, according to Hybrid 2 and Hybrid 4 impact specimens with ballistic impact energy absorption of 95.17 J and 95.15 J, respectively. Moreover, the results indicated that using the combination of carbon and glass is more efficient to in the central layers. Third, in accordance with Hybrid 1 with ballistic impact energy absorption of 94.36 J, using the carbon fibre is not recommended at the last layer.

## Figures and Tables

**Figure 1:** Ballistic test setup according to NIJ Standard 0108.01 [5].

**Figure 2:** (a) Gun equipment [9] and (b) gas gun [10].

**Figure 3:** Gas gun tunnel for conducting the ballistic impact test [12].

**Figure 4:** Schematic of the cylindrical AISI 4340 Steel pellet [17, 18].

**Figure 5:** Process of penetration of pellet into the specimens [17, 18].

**Figure 6:** Comparison of the specimens' weight losses' percentages after ballistic impact.

**Figure 7:** Postimpact images of damaged specimens' profiles. (a) Impact-induced damage profile viewed from the front face and (b) impact-induced damage profile viewed from the back face.

**Figure 8:** The perimeter of the impacted zones.

**Figure 9:** Comparing the amount of energy absorption in the specimens of 182 m/s as the initial velocity.

**Figure 10:** Comparison of the energy absorption and different final velocities of six specimens at 182 m/s as the initial velocity.

**Figure 11:** Percentage change of the COR.

**Table 1:** Fabricated composite plates were divided into five groups (from top surface to bottom surface) [17, 18].

HYBRID 1	HYBRID 2	HYBRID 3	HYBRID 4	HYBRID 5
Kevlar	Glass	Kevlar	Glass	Kevlar
Carbon	Carbon	Glass	Kevlar	Carbon
Glass	Kevlar	Carbon	Carbon	Glass
Kevlar	Carbon	Glass	Carbon	Glass
Glass	Kevlar	Carbon	Glass	Carbon
Carbon	Glass	Kevlar	Kevlar	Kevlar

**Table 2:** Final velocity and energy absorption of the specimens.

Specimen	Final velocity (m/s)	Ballistic energy absorption (J)
Hybrid 1	14.36	94.36
Hybrid 2	4.47	95.17
Hybrid 3	8.76	95.01
Hybrid 4	5.28	95.15
Hybrid 5	8.21	95.04
Carbon	26.87	93.16

*Initial velocity is 182 m/s.
